# Protective Effect of Luteolin on D-Galactosamine (D-Gal)/Lipopolysaccharide (LPS) Induced Hepatic Injury by in Mice

**DOI:** 10.1155/2021/2252705

**Published:** 2021-07-28

**Authors:** Yiwei Pu, Zhaocong Yang, Xuming Mo

**Affiliations:** Department of Cardiothoracic Surgery, Children's Hospital of Nanjing Medical University, Nanjing, China

## Abstract

To observe the effects of luteolin on galactosamine (D-Gal)/lipopolysaccharide (LPS) induced liver injury in mice. Male C57BL/6 mice were randomly divided into 4 groups: normal control group, D-GaI/LPS group, D-GaI/LPS + luteolin (Lu, 20 mg/kg), and D-GaI/LPS + luteolin (Lu, 40 mg/kg). Mice in the normal control group and D-GaI/LPS group were given distilled water while other groups were given drugs in 7 days by gavage. 4 hours after the continuous administration, Gal (700 mg/kg) and LPS (10 mg/kg) were injected intraperitoneally. Mice in the normal control group were given the same volume of vegetable oil solution. 24 h after the establishment of the mice model, blood and liver samples were collected. Hematoxylin (HE) staining was used to observe the changes of hepatic histopathology. Alanine aminotransferase (ALT) and glutamic oxalacetic transaminase (AST) in serum, interleukin-6 (IL-6), interleukin-1*β* (IL-1*β*), and tumor necrosis factor (TNF-*α*) were measured by related kits. Western blotting was used to demonstrate the expression levels of related inflammation proteins. Lu significantly reduced levels of proinflammatory cytokines including interleukin-6 (IL-6), interleukin-1*β* (IL-1*β*), and tumor necrosis factor-*α* (TNF-*α*) in serum and liver. Lu restored the pathological changes after galactosamine (D-Gal)/lipopolysaccharide (LPS) treatment. In addition, Lu regulated proteins levels of the NLRP3/NF-*κ*B pathway in liver. Lu exhibited therapeutical effects on D-GaI/LPS induced liver injury in mice which might be related to the regulation of the NLRP3/NF-*κ*B pathway.

## 1. Introduction

Acute hepatic failure (AFT) is a serious clinical syndrome, which is the result of a large number of hepatocyte deaths [1]. The prognosis of acute liver failure is very poor, and there is no effective treatment unless liver transplantation. Drug-induced liver injury (DILI) is a major cause of AFT which is one of the leading causes for liver transplantation [2]. The liver injury caused by simultaneous injection of d-galactosamine (d-gal) and lipopolysaccharide (LPS) has been widely used to study the pathogenesis of AFT [3–5]. Although it is well known that hepatocyte is the main target cell of AFT, hepatocyte (such as macrophages and neutrophils) has an inflammatory reaction. The mechanism of liver injury induced by d-gal/LPS is not completely clear [6]. Therefore, it is urgent to study the mechanism of AFT and the drug treatment.

D-galactosamine is a classic model for the preparation of acute liver injury. The main pathogenic component of bacterial lipopolysaccharide gram-negative bacteria can cause systemic inflammatory response syndrome, which can lead to acute liver injury and multiple organ failure. D-galactosamine (D-gal) can increase the sensitivity of mice to lipopolysaccharide and aggravate the lethal effect of lipopolysaccharide. Therefore, D-galactosamine (D-gal) and lipopolysaccharide (LPS) were used to replicate the liver injury model of mice in this experiment.

NLRP3 inflammasome (Nucleotide-binding and oligomerization domain-like receptors3 inflammasome), a newly discovered pattern recognition receptor (PRRs), is an important membership of host immune defense system, including NLRP3 molecules, ligand molecules ASC (apoptosis-associated spec-like protein), and procaspase-1, which is composed of three molecules whose binding state regulates the activity of NLRP3 inflammasome corpuscles [7]. In the liver, NLRP3 inflammasome corpuscles were mainly expressed in hepatocyte. NLRP3 inflammasome consists of NLRP3, ASC, and caspase-1. Caspase-1 is crucial to the conversion of IL-1*β* immature type to active type. The response of NLRP3 to stimulus requires NF-*κ*B signaling.

Luteolin (3′, 4′, 5,7–tetrahydroxyflavone, Lu), a common flavonoid found in various plants, is reported to have various pharmacological correlations, including free radical scavenging anticancer and anti-inflammatory activities [8, 9]. However, there are still few studies on whether Lu is beneficial for acute liver failure. Luteolin has also been shown to exhibit a therapeutic effect on liver injury induced by tetrachloromethane (CCl4) [10], ethanol [11], or acetaminophen [12] in mice. Therefore, our research is aimed at evaluating the effects of Lu on acute liver failure and exploring its possible mechanism.

## 2. Materials and Methods Reagents and Kits

Lu was obtained from Sigma-Aldrich (Saint Louis, MO, USA). Gal and LPS were obtained from Sigma Aldrich (St. Louis, USA). Interleukin- (IL-) 6, IL-1*β*, and tumor necrosis factor- (TNF-) *α* enzyme-linked immunosorbent assay (ELISA) kits were obtained from Elabscience (Wuhan, China). Primary antibodies were purchased from Cell Signaling Technology. The commercial kits of alanine aminotransferase (ALT) and glutamic oxalacetic transaminase (AST) were purchased from Jiancheng Bioengineering Institute (Nanjing, China).

### 2.1. Animals

60 male C57BL/6 mice (20-22 g) were purchased from the experimental animal center of Nantong University, Certificate No. SCXK (Su) 2012-0001. Animal welfare and experimental procedures strictly abide by the ethical guidelines of the National Institutes of Health and were approved by the Institutional Animal Research Committee of Nanjing Medical University.

### 2.2. Experimental Procedure

60 male C57BL/6 mice were randomly divided into 4 groups, 15 in each group: control group, D-GaI/LPS group, D-GaI/LPS + Lu (20 mg/kg), and D-GaI/LPS + Lu (20 mg/kg) (40 mg/kg). Lu (20, 40 mg/kg) was given continuously by gastric perfusion for 7 days, while the control group and the D-GaI/LPS group were given the same amount of distilled water. Four hours after the last administration, D-GaI (700 mg/kg) and LPS (10 mg/kg) were injected intraperitoneally to mice, while the control group was injected intraperitoneally with equal volume of solvent. After 24 h, the animals were sacrificed to collect the blood and liver tissue.

### 2.3. HE Staining of Liver Tissue

C57BL/6 mice liver tissue was fixed in 4% neutral formalin solution. The liver tissue was then embedded in paraffin and cut into 4 mm thick slices. Finally, hematoxylin-eosin staining (HE staining) was performed to observe the histopathological changes of the liver under optical microscope.

### 2.4. Biochemical Assays in Serum

The levels of ALT and AST were determined by commercial kits according to the manufacturer's instructions.

### 2.5. Determination of Cytokines in Serum and Liver

The contents of IL-1*β*, IL-6, and TNF-*α* in serum and liver of mice of each group were detected according to ELISA kit instructions.

### 2.6. Determination of NLRP3/NF-*κ*B-Related Protein in Liver

The total protein in liver tissue of mice in each group was extracted with RIPA lysate, centrifuged at 12,000 rpm for 15 minutes, and supernatant was collected. The BCA kit was used to quantify the proteins of each group. The protein samples of each group were subjected to SDS-polyacrylamide gel electrophoresis and then transferred to PVDF membrane. Then, the PVDF membrane was placed in 5 % skimmed milk and sealed for 2 h. After 2 hours of sealing, PVDF membrane was placed in the corresponding primary antibody and incubated overnight at 4°C. The next day was washed 4 times with TBST for 8 min each time. Then, the PVDF membrane was placed in the second antibody solution and incubated for 2 h at room temperature in a shaking table. PVDF membrane was removed and washed 4 times with TBST for 8 min each time. The gel imaging system was used to expose and scan the bands to analyze the gray value of each band.

### 2.7. Immunohistochemistry

The expressions of NLRP3 and p-NF-*κ*BP65, in the liver of mice, were detected by immunohistochemical method. In short, liver tissue was fixed with 4 % paraformaldehyde (PFA), embedded in paraffin, and sliced. Paraffin sections were dewaxed in xylene and absolute ethanol, microwave in sodium citrate buffer, and washed with PBS. Endogenous peroxidase activity was blocked by 3 % hydrogen peroxide for 20 min. Each sample was blocked with 5% goat serum for 20 minutes and then treated with primary antibodies NLRP 3 (1 : 200) and p-NF-*κ*Bp65 (1 : 200), overnight at 4°C. The next day, after washing with PBS for 3 times, each sample was treated with goat anti-rabbit IgG secondary antibody for 20 min, then the horseradish enzyme-labeled streptavidin working solution was incubated for 20 min, and washed with PBS for 3 times. Then stained with 3-3′ diaminobenzidine (DAB) and then stained with hematoxylin. After dehydration and drying, the slices were fixed with neutral glue and observed under a microscope.

### 2.8. Statistical Analysis

All the experimental data were expressed as mean standard deviation, and one-way ANOVA was performed with statistical software. *P* < 0.05 showed that the difference was statistically significant.

## 3. Results

### 3.1. Effects of Lu on ALT and AST in Liver Injury Mice Induced by D-GaI/LPS

As is shown in Figure 1, compared with the control group, the contents of ALT and AST in the model group were significantly increased after injection of D-GaI/LPS. Compared with the model group, Lu (20, 40 mg/kg) could significantly reduce ALT and AST contents.

### 3.2. Effects of Lu on Cytokines in Serum of D-GaI/LPS-Induced Liver Injury Mice

As is shown in Figure 2, compared with the control group, the levels of IL-1*β*, IL-6, and TNF-*α* in the serum of mice in the model group were significantly increased. Compared with the model group, the contents of IL-1*β*, IL-6, and TNF-*α* in Lu (20, 40 mg/kg) groups were significantly lower than those in the model group.

### 3.3. Effects of Lu on Cytokines in Liver of D-GaI/LPS-Induced Liver Injury Mice

As is shown in Figure 3, compared with the control group, the levels of IL-1*β*, IL-6, and TNF-*α* in the liver of mice in the model group were significantly increased. Compared with the model group, the contents of IL-1*β*, IL-6, and TNF-*α* in Lu (20, 40 mg/kg) groups were significantly lower than those in the model group.

### 3.4. Effect of Lu on Liver Tissue Pathological Changes in D-GaI/LPS-Induced Liver Injury Mice

As shown in Figure 4, the liver tissue structure of the mice in the control group is normal and the cell morphology is normal. In the model group, the liver tissue structure was abnormal, liver cells were denatured, and inflammatory cells infiltrated. Compared with the model group, the liver structure and hepatocyte morphology in Lu (20, 40 mg/kg) groups were basically normal, and inflammatory cell infiltration was reduced.

### 3.5. Effect of Lu on the Expression of NLRP3/NF-*κ*B Pathway Protein in Liver of D-GaI/LPS-Induced Liver Injury Mice

As shown in Figure 5, compared with the group, the expression of NLRP3, ASC, Caspapse-1, IL-1*β*, p-I*κ*B*α*, and p-NF-*κ*Bp65 protein in the model group were significantly increased. Compared with the model group, the expression of NLRP3, ASC, Caspapse-1, IL-1*β*, p-I*κ*B*α*, and p-NF-*κ*Bp65 protein in liver tissue of mice in Lu (20, 40 mg/kg) groups was significantly decreased.

### 3.6. Effect of Lu on the Expression of NLRP3 and p-NF-*κ*Bp65 in Liver of D-GaI/LPS-Induced Liver Injury Mice by Immunohistochemistry

As shown in Figure 6, compared with the control group, the expression of NLRP3 and p-NF-*κ*Bp65 in the model group was significantly increased. Compared with the model group, the expression of NLRP3 and p-NF-*κ*Bp65 in liver tissue of mice in Lu (20, 40 mg/kg) groups was significantly decreased.

## 4. Discussion

The liver injury model induced by D-GaI/LPS was used in this study. It was found that Lu could significantly reduce ALT and AST activities and reduce the content of proinflammatory cytokines such as IL-1*β*, IL-6, and TNF-*α* in serum and liver induced by D-GaI/LPS. The results of western blot suggest that Lu may have protective effects on liver injury via inhibiting NLRP3/NF-*κ*B pathway.

Alanine aminotransferase (ALT) and aspartate aminotransferase (AST) are both present in liver. When the hepatocyte membrane is damaged or the cell is necrotic, the enzymes entering the supernatant increase. ALT and AST activities in the supernatant can sensitively reflect the degree of hepatocyte injury [13]. In the early stage of acute liver injury, ALT change is the most sensitive, and it is the main item to diagnose hepatocyte parenchymal damage. ALT level is often parallel to the severity of the disease. However, when liver injury occurs, AST increases to a higher level than ALT. At that time, AST is the main indicator of the degree of liver injury. ALT mainly exists in hepatocyte plasma, while AST exists in hepatocyte plasma and is distributed in mitochondria. AST and ALT are commonly used indicators of liver fibrosis. Previous studies have shown that the administration of D-GaI/LPS distinctly increased the activities of ALT and AST. However, pretreatment with flavonoid strikingly reduced AST and ALT activities [14]. Our study showed the change of serum enzyme of ALT and AST levels was consistent with the above results.

Inflammatory reaction is one of the important causes of liver injury. Inhibition of inflammatory reaction can improve the symptoms of liver injury [15]. Therefore, anti-inflammatory protection of liver cells is crucial in the treatment of liver injury. After the occurrence of liver parenchymal injury, hepatocyte is activated to release more inflammatory mediators IL-1*β*, IL-6, and TNF-*α*, which could influence HSC and Kuffer cells. It forms positive feedback regulation, resulting in more cytokines and aggregation, thus, promoting the development of liver injury [16]. The contents of IL-1*β*, IL-6, and TNF-*α* in liver injury serum were significantly higher than those in the normal control group and gradually increased with the aggravation of liver injury. IL-1*β*, IL-6, and TNF-*α* participate in the whole process of the occurrence and development of acute liver injury [17]. In this study, the expression of IL-1*β*, IL-6, and TNF-*α* in serum and liver was significantly increased under the stimulation of D-GaI/LPS. Lu could inhibit the production and release of inflammatory factors in serum and liver of mice with liver injury induced by D-GaI/LPS. Park et al. found that luteolin administration significantly ameliorated the increased TNF-*α* production and COX-2 expression in GalN/LPS-induced hepatitic ICR mice [18]. Attiq et al. reported Lu abrogates the LPS-induced inflammatory responses in human plasma, especially decreased the expression of IL-1*β* and IL-6 [19].

TNF-*α* secretion is regulated by The TLR4/NF-*κ*B signaling pathway in liver [20, 21]. NF-*κ*B belongs to Rel protein family, in which the heterodimer composed of p65 and p50 is a trimer formed by combining NF-*κ*B with I*κ*B*α* in resting state and exists in cytoplasm in inactive form. NF-*κ*B was reported regulating the inflammation in CCl4 exposure-induced hepatitis to ameliorate liver injury [22, 23]. When stimulated by external signals, it activates a series of protein kinases, such as NLRP3 inflammasome, thus, mediating inflammatory reactions [24]. LPS could cause the expression and activation of NLRP3, while luteolin treatment could inhibit the expression and activation of NLRP3 [25]. There was no report that luteolin is effective in LPS-induced liver failure through NLRP3/NF-*κ*B inflammatory pathway. NLRP3 inflammasome is a protein complex composed of receptor protein, apoptosis-associated specific-like protein (CARD), ASC, and effector molecule pro-caspase-1. It forms a cysteine proteolytic enzyme (Caspase) self-shearing that can lead to inflammatory aspartic acid specificity. The latter causes host inflammatory response by activating proinflammatory factors IL-1*β* and IL-18. The existing literature has proved the inflammatory regulatory effect of the NLRP3/NF-*κ*B pathway in the course of liver injury [26]. This study proves that Lu can significantly reduce the increased production of NLRP3, ASC, Caspapse-1, IL-1*β*, p-I*κ*B*α*, and p-NF-*κ*Bp65 caused by D-GaI/LPS.

## 5. Conclusion

To sum up, our experiment shows that Lu can improve the liver injury induced by D-GaI/LPS in mice, and the effect may be through NLRP3/NF-*κ*B signal pathway, and the specific mechanism needs further study.

## Figures and Tables

**Figure 1:** Effects of Lu on ALT and AST in liver injury mice induced by D-GaI/LPS. The values are presented as the mean ± standard deviation. ^∗^*P* < 0.05 compared to the D-GaI/LPS group; ^∗∗^*P* < 0.01 compared to the D-GaI/LPS group; ^#^*P* < 0.01 compared to the control group, ^##^*P* < 0.01 compared to the control group.

**Figure 2:** Effects of Lu on cytokines in serum of D-GaI/LPS-induced liver injury mice. The values are presented as the mean ± standard deviation. ^∗^*P* < 0.05 compared to the D-GaI/LPS group; ^∗∗^*P* < 0.01 compared to the D-GaI/LPS group; ^#^*P* < 0.01 compared to the control group, ^##^*P* < 0.01 compared to the control group.

**Figure 3:** Effects of Lu on cytokines in liver of D-GaI/LPS-induced liver injury. The values are presented as the mean ± standard deviation. ^∗^*P* < 0.05 compared to the D-GaI/LPS group; ^∗∗^*P* < 0.01 compared to the D-GaI/LPS group; ^#^*P* < 0.01 compared to the control group, ^##^*P* < 0.01 compared to the control group.

**Figure 4:** Effect of Lu on liver tissue pathological changes in D-GaI/LPS-induced liver injury mice (×200). The values are presented as the mean ± standard deviation. ^∗^*P* < 0.05 compared to the D-GaI/LPS group; ^∗∗^*P* < 0.01 compared to the D-GaI/LPS group; ^#^*P* < 0.01 compared to the control group, ^##^*P* < 0.01 compared to the control group.

**Figure 5:** Effect of Lu on the expression of NLRP3/NF-*κ*B pathway protein in liver of D-GaI/LPS-induced liver injury mice. The values are presented as the mean ± standard deviation. ^∗^*P* < 0.01 compared to the D-GaI/LPS group; ^∗∗^*P* < 0.01 compared to the D-GaI/LPS group; ^#^*P* < 0.01 compared to the control group, ^##^*P* < 0.01 compared to the control group.

**Figure 6:** Effect of Lu on the expression of NLRP3 and p-NF-*κ*Bp65 in liver of D-GaI/LPS-induced liver injury mice by immunohistochemistry. The values are presented as the mean ± standard deviation. ^∗^*P* < 0.05 compared to the D-GaI/LPS group; ^∗∗^*P* < 0.01 compared to the D-GaI/LPS group; ^#^*P* < 0.01 compared to the control group, ^##^*P* < 0.01 compared to the control group.

## Data Availability

The raw data could be accessed by contact the corresponding author if necessary.

## References

[1] Hoofnagle J. H., Carithers R. L., Shapiro C., Ascher N. (1995). Fulminant hepatic failure: summary of a workshop. *Hepatology*.

[2] Fernandez-Checa J. C., Bagnaninchi P., Ye H. (2021). Advanced preclinical models for evaluation of drug induced liver injury - consensus statement by the european drug-induced liver injury network [pro- euro-dili-net]. *Journal of Hepatology*.

[3] Nakama T., Hirono S., Moriuchi A. (2001). Etoposide prevents apoptosis in mouse liver with D-galactosamine/lipopolysaccharide-induced fulminant hepatic failure resulting in reduction of lethality. *Hepatology*.

[4] Kuhla A., Eipel C., Siebert N., Abshagen K., Menger M. D., Vollmar B. (2008). Hepatocellular apoptosis is mediated by TNF*α*-dependent Fas/FasLigand cytotoxicity in a murine model of acute liver failure. *Apoptosis*.

[5] Eipel C., Kidess E., Abshagen K. (2007). Antileukoproteinase protects against hepatic inflammation, but not apoptosis in the response of D-galactosamine-sensitized mice to lipopolysaccharide. *British Journal of Pharmacology*.

[6] Shakil A. O., Kramer D., Mazariegos G. V., Fung J. J., Rakela J. (2000). Acute liver failure: clinical features, outcome analysis, and applicability of prognostic criteria. *Liver Transplantation*.

[7] Lee W. M. (1993). Acute liver failure. *The New England Journal of Medicine*.

[8] Mignon A., Rouquet N., Fabre M. (1999). LPS challenge in D-galactosamine-sensitized mice accounts for caspase-dependent fulminant hepatitis, not for septic shock. *American Journal of Respiratory and Critical Care Medicine*.

[9] Imran M., Rauf A., Abu-Izneid T. (2019). Luteolin, a flavonoid, as an anticancer agent: a review. *Biomedicine & Pharmacotherapy*.

[10] Domitrović R., Jakovac H., Milin C., Radošević-Stašić B. (2009). Dose- and time-dependent effects of luteolin on carbon tetrachloride-induced hepatotoxicity in mice. *Experimental and Toxicologic Pathology*.

[11] Liu G., Zhang Y., Liu C. (2014). Luteolin alleviates alcoholic liver disease induced by chronic and binge ethanol feeding in mice. *The Journal of Nutrition*.

[12] Tai M., Zhang J., Song S. (2015). Protective effects of luteolin against acetaminophen-induced acute liver failure in mouse. *International Immunopharmacology*.

[13] Kaufman R. J. (1999). Stress signaling from the lumen of the endoplasmic reticulum: coordination of gene transcriptional and translational controls. *Genes & Development*.

[14] He Y., Xia Z., Yu D. (2019). Hepatoprotective effects and structure-activity relationship of five flavonoids against lipopolysaccharide/d-galactosamine induced acute liver failure in mice. *International Immunopharmacology*.

[15] Ron D., Walter P. (2007). Signal integration in the endoplasmic reticulum unfolded protein response. *Nature Reviews. Molecular Cell Biology*.

[16] Xu C., Bailly-Maitre B., Reed J. C. (2005). Endoplasmic reticulum stress: cell life and death decisions. *The Journal of Clinical Investigation*.

[17] Rao R. V., Ellerby H. M., Bredesen D. E. (2004). Coupling endoplasmic reticulum stress to the cell death program. *Cell Death and Differentiation*.

[18] Park C. M., Song Y. S. (2019). Luteolin and luteolin-7-O-glucoside protect against acute liver injury through regulation of inflammatory mediators and antioxidative enzymes in GalN/LPS-induced hepatitic ICR mice. *Nutrition Research and Practice*.

[19] Attiq A., Jalil J., Husain K., Mohamad H. F., Ahmad A. (2021). Luteolin and apigenin derived glycosides from *Alphonsea elliptica* abrogate LPS-induced inflammatory responses in human plasma. *Journal of Ethnopharmacology*.

[20] Zhao S., Jiang J., Jing Y. (2020). The concentration of tumor necrosis factor-*α* determines its protective or damaging effect on liver injury by regulating Yap activity. *Cell Death & Disease*.

[21] Wang H., Wei X., Wei X. (2020). 4-hydroxybenzo[d]oxazol-2(3H)-one ameliorates LPS/D-GalN-induced acute liver injury by inhibiting TLR4/NF-*κ*B and MAPK signaling pathways in mice. *International Immunopharmacology*.

[22] Seif M., Deabes M., el-Askary A. (2021). Ephedra sinica mitigates hepatic oxidative stress and inflammation via suppressing the TLR4/MyD88/NF-*κ*B pathway in fipronil-treated rats. *Environmental Science and Pollution Research International*.

[23] Dai C., Li H., Wang Y., Tang S., Velkov T., Shen J. (2021). Inhibition of oxidative stress and ALOX12 and NF-*κ*B pathways contribute to the protective effect of baicalein on carbon tetrachloride-induced acute liver injury. *Antioxidants (Basel)*.

[24] Ning Z. W., Luo X. Y., Wang G. Z. (2017). MicroRNA-21Mediates angiotensin II-induced liver fibrosis by activating NLRP3 Inflammasome/IL-1*β* AxisviaTargetingSmad7andSpry1. *Antioxidants & Redox Signaling*.

[25] Wang X., Wang L., Dong R. (2021). Luteolin ameliorates LPS-induced acute liver injury by inhibiting TXNIP-NLRP3 inflammasome in mice. *Phytomedicine*.

[26] Wu X., Zhang F., Xiong X. (2015). Tetramethylpyrazine reduces inflammation in liver fibrosis and inhibits inflammatory cytokine expression in hepatic stellate cells by modulating NLRP3 inflammasome pathway. *IUBMB Life*.

